# Blasting Law of Liquid CO_2_ Phase Change in Coal Mine Based on Numerical Simulation

This article has been retracted.

**DOI:** 10.1155/2022/6866925

**Published:** 2022-08-27

**Authors:** Bo Fang

**Affiliations:** College of Safety Science & Engineering, Liaoning Technical University, Fuxin 123000, China

## Abstract

In order to obtain the best CO_2_ blasting drilling efficiency and improve the gas permeability coefficient of the coal seam in the mining area, a research method of liquid CO_2_ phase change blasting in the coal seam based on electrochemical numerical simulation is proposed. In this paper, the electrochemical numerical simulation of coalbed methane caused by liquid CO_2_ phase change blasting is studied through theoretical analysis, the antireflection mechanism of liquid carbon dioxide gas explosion on broken coal seam is obtained, and the initial fracture length of coal body caused by gas explosion stress wave is deduced by the mathematical model. A method for improving CBM desorption with nonmechanical coal was proposed, namely, a method for electrochemically strengthening CBM desorption. A comprehensive theory and application system of liquid carbon dioxide phase change gas explosion and anti-reflection technology are established by combining theoretical analysis, experimental research, and numerical simulation with field industrial comparative experiment. According to the gas tracing method, the precise measurement of the working face shows that the impact radius of the collision caused by the explosion of the liquid carbon dioxide phase change gas is 2 m. Gas emissions increased the emissions of coal seam drilling in the affected areas by 4 to 8 times, and the gas emission attenuation coefficient decreased from 0.76 times to 0.93 times. The carbon dioxide phase change gas cracking theory and antireflection theory and their application technology system are systematically studied. The research shows that the liquid carbon dioxide phase transfer gas blasting and infiltration technology is not limited by the geological conditions of the coal seam and has the characteristics of high efficiency and inherent climate. In view of the wide area of coal mines and the harsh geological conditions of coal seams, carbon dioxide phase change gas-induced cracking antireflection technology has application prospects and expandability.

## 1. Introduction

In coal mine underground mining, industrial accidents caused by gas account for about 30% ∼ 40%. Therefore, gas drainage is usually regarded as the main technical measure to prevent major gas disasters and accidents in coal mine. In recent years, with the rapid development of blasting machines, the application of blasting has become more and more extensive, which makes it more difficult to improve and mature the blasting technology [1]. As shown in Figure 1, the safety measures have to be taken at present. In addition, coal is a kind of soft rock. Due to its special structure and the existence of gas in coal, there is a certain connection and difference between coal blasting and rock blasting. In order to improve oil discharge, it is first necessary to improve the permeability of exhaust gas and carbon monoxide, which requires further research on the blasting process of coal under gas [2]. The application of blasting technology in coal mining has a long history. Nowadays, no matter the excavation of roadway or the crushing of rock mass and coal body, blasting technology is not necessary. However, whether hydraulic fracturing blasting technology, preblasting weakening technology of hard top coal, deep hole loose blasting technology, or blasting construction technology in other coal bodies, the blasting mechanism of coal body needs to be used. However, although many scholars have studied the rock cylindrical charge blasting, the research on the blasting mechanism is only in the initial stage, and the relevant research results are less [3]. Accordingly, the blasting technology is also difficult to get a breakthrough development, which cannot meet the needs of actual coal mine production.

## 2. Literature Review

Zhang et al. and others believe that with the improvement of coal mine mechanization, the mining depth of the mine is deeper and deeper, resulting in the increasing ground stress of the coal seam, the reduction of permeability coefficient, and the gradual reduction of gas drainage efficiency, which seriously affects the connection of mine mining [4]. In order to improve the permeability coefficient and smoke exhaust efficiency of coal seams, Ma and Du have developed several methods to improve the permeability of coal seams in recent years: high squeezing liquids and deep priority—split blasting, hydraulic measurement, and other technologies. However, these methods have problems such as imperfect technical conditions and processes, unsafe factors, or causing coal outbursts, resulting in unsatisfactory effect of coal seam enhancement [5]. In view of this phenomenon, scientific researchers put forward the liquid CO_2_ cracking and permeability enhancement technology. Yu and others analyzed the pressure time history change of high-pressure gas in the main pipe of the cracking cylinder during liquid CO_2_ blasting based on damage mechanics and aerodynamics. The field test found that the permeability coefficient of coal seam after blasting increased by 17.49 ∼ 22.76 times [6]; OLLIS, T. and others carried out tests in a coal mine and obtained that after the implementation of CO_2_ controllable phase change cracking and outburst prevention technology in the heading face, compared with the conventional intensive emission borehole outburst elimination technology, the CO_2_ controllable phase change cracking and outburst prevention technology has less gas desorption index △h2 by 50%, and the gas drainage volume is increased by twice, significantly improving the excavation speed [7]. CO_2_ phase transfer fracturing blasting technology is used in high gas and low-permeability coal seams. It is determined that when the blasting is not CO_2_ blasting, the blasting distance is 5 m, and the blasting distance is 7.5 m, the permeability enhancement effect of the coal seam is the best [8]. That is to say, it solves the problem of large gas volume and excessive oblique oil volume affecting the speed during the mining of concrete working face, and rapidly improves the decomposition and permeability of liquid CO_2_. With the help of theoretical analysis and numerical simulation, the liquid CO_2_ cracking and anti-reflection technology is studied, and the field test is carried out to compare and analyze the gas extraction effect before and after blasting, so as to achieve the purpose of high-efficiency recovery of low permeability coal seam. Permeable seam [9]. Zhang et al. and others said that doing a good job in gas drainage is the fundamental measure to reduce coal mine gas disasters. Gas extraction can not only effectively prevent coal mine gas accidents but also reduce environmental pollution caused by gas discharged into the air [10]. Jin and Yang and others obtained through research that the greenhouse effect of gas is about 21 times that of carbon dioxide, and the ability to penetrate the ozone layer is 7 times higher. Therefore, accelerating the extraction and utilization of gas and transforming harmful gas into useable energy is a major trend in the energy field [11]. Lu et al. and others said that in order to protect the living environment of mankind, the development and utilization of coalbed methane is regarded as an energy plan in the new century all over the world, which will inevitably promote the rapid development of China's coalbed methane mining industry [12]. Xie et al. and others believe that the main problem at present is the low permeability of coal seam, and the adsorbed gas is difficult to be fully decomposed and absorbed, which brings great difficulties to the development of coalbed methane. How to improve the desorption rate and permeability of gas in coal seams, how to improve the extraction technology, and how to effectively solve the problem of low gas extraction rate have become the focus of CBM mining research [13].

## 3. Methods

### 3.1. Analysis of Crack Propagation in Coal Seam Explosion by Liquid Carbon Dioxide Phase Change Gas Explosion

According to the elastic mechanics theory, the stress state at any point around the borehole wall of the coal seam permeability enhancement target is shown in

(1) $$\begin{array}{c} \left\{\begin{array}{c} \sigma_{rr\text{geo}}=-\frac{\sigma_{yy\text{geo}}}{2}\left[\left(1+K\right)\left(1-\frac{r_{b}^{2}}{r^{2}}\right)-\left(1-K\right)\left(1-\frac{4r_{b}^{2}}{r^{2}}+\frac{3r_{b}^{2}}{r^{4}}\cos2\theta \right)\right],\\ \sigma_{\theta \theta \text{geo}}=-\frac{\sigma_{yy\text{geo}}}{2}\left[\left(1+K\right)\left(1-\frac{r_{b}^{2}}{r^{2}}\right)+\left(1-K\right)\left(1-\frac{4r_{b}^{2}}{r^{2}}+\frac{3r_{b}^{2}}{r^{4}}\cos2\theta \right)\right],\\ \sigma_{r\theta \text{geo}}=-\frac{\sigma_{yy\text{geo}}}{2}\left[\left(1-K\right)\left(1+\frac{r_{b}^{2}}{r^{2}}+\frac{3r_{b}^{2}}{r^{4}}\sin2\theta \right)\right], \end{array}\right. \end{array}$$

where *σ*_*rr*geo_, *σ*_*θθ*geo_, and *σ*_*rθ*geo_ are the stress at each location of the fractured skeleton in polar coordinates, respectively; *σ*_*yy*geo_ is the vertical stress component; K is the lateral pressure coefficient of in-situ stress in horizontal direction; and *θ* is the angle between the horizontal direction and the polar coordinates. It has been shown that gas peaks and waves from carbon dioxide phase breakup change the appearance of gas, and they are shown in

(2) $$\begin{array}{c} P_{g}=\frac{1}{8}\rho_{0}D^{2}{\left(\frac{d_{1}}{d_{2}}\right)}^{6}{\left(\frac{I_{1}}{I_{2}}\right)}^{3}, \end{array}$$

(3) $$\begin{array}{c} P_{\delta }=\frac{1}{8}\rho_{0}D^{2}{\left(\frac{d_{1}}{d_{2}}\right)}^{6}{\left(\frac{I_{1}}{I_{2}}\right)}^{3}\cdot n, \end{array}$$

where *p*_*g*_ and *p*_*δ*_ are the high pressure and explosion waves formed by the explosion of carbon dioxide phase change fuel, respectively; *p*_*o*_ is the density of carbon dioxide; *D* is the diffusion rate of liquid carbon dioxide phase change; *d*_1_ and *d*_2_ are the diameters of the cracker and the cracker borehole, respectively, *I*_1_ and *I*_2_ are the depths of the cracker gas storage chamber and the cracker borehole, respectively, and N is the increment coefficient, which is generally taken as 8 ∼ 11 [14].

The shock wave generated by the gas explosion attenuates rapidly in the coal seam around the borehole. The relationship between the gas explosion pressure and the propagation distance is shown in the following equation:

(4) $$\begin{array}{c} P\left(r\right)=P_{\delta }{\left(\bar{r}\right)}^{-\alpha }, \end{array}$$

where $\bar{r}=r/r_{b}$, *r*_*b*_ is the radius of the borehole fracture; *r* is the distance from the center of the borehole fracture; *α* is the attenuation coefficient of gas explosion shock wave, which is taken as 3.

The relationship between the wave velocity of the gas explosion wave in the coal and the electric field velocity is shown in the following equation:

(5) $$\begin{array}{c} D=a+bv, \end{array}$$

where *V* is the velocity of the wavefront particle; *a* and *b* are experimentally measured values, respectively [15].

Gas radiation waves propagate in the coal seam and decay slowly into stress waves. The velocity of the stress wave is *c*_*p*_. According to the conservation of energy, the maximum energy velocity wave propagating to the compression edge can be expressed by :

(6) $$\begin{array}{c} P_{m}=\rho_{c}c_{p}v_{r}. \end{array}$$

A quick perception of coal and rock associated with the collision edge of a gas explosion can be presented according to the following equation:

(7) $$\begin{array}{c} v_{r}=\frac{\left(c_{p}-a\right)}{b}. \end{array}$$

The radius of the near zone of phase change gas explosion can be obtained from equation (4)–(7), as shown in the following equation:

(8) $$\begin{array}{c} r_{c}=r_{b}{\left[\frac{b\left(p_{\delta }\right)}{\rho_{c}c_{p}\left(c_{p}-a\right)}\right]}^{1/3}. \end{array}$$

Therefore, the crack propagation length *L*_1_ formed in the gas explosion crushing area is shown in the following equation:

(9) $$\begin{array}{c} L_{1}=r_{c}-r_{b}=r_{b}\left[{\left[\frac{bp_{s}}{\rho_{c}c_{p}\left(c_{p}-a\right)}\right]}^{1/3}-1\right]. \end{array}$$

Previous studies have shown that the stress equivalent equation is represented by the following equation:

(10) $$\begin{array}{c} \alpha =\left[\frac{3-\mu }{\left(2-\mu \right)}\right]. \end{array}$$

According to the Poisson results, the expression of the peak value of the tangential tensile stress in the fracture stress wave region of the bone region is shown in the following equation:

(11) $$\begin{array}{c} \sigma_{\theta \theta \max}=P_{m}\left[\frac{\mu }{1-\mu }{\left(\frac{r_{b}}{r}\right)}^{\alpha }\right]. \end{array}$$

The total tangential stress at any point of the coal body in the fracture area can be expressed as shown in the following equation:

(12) $$\begin{array}{c} \sigma_{\theta \theta 1}=\sigma_{\theta \theta \max}+\Sigma_{\theta \theta \text{geo}}=P_{m}\left[\frac{\mu }{1-\mu }{\left(\frac{r_{b}}{r}\right)}^{\alpha }\right]+\sigma_{\theta \theta \text{geo}}. \end{array}$$

The dynamic tensile strength *σ*_d*t*_ of coal is replaced by *σ*_*θθ*1_, and the expression of the expansion range of radial crack caused by the stress wave after phase change gas explosion is obtained, as shown in the following equation:

(13) $$\begin{array}{c} r_{2}=r_{b}{\left(\frac{\mu P_{m}}{\left(1-\mu \right)\left(\sigma_{dt}-\sigma_{\theta \theta geo}\right)}\right)}^{1/\alpha }. \end{array}$$

The initial burst duration representing the coal explosion caused by the liquid carbon dioxide phase transition combustible stress wave is given by the following equation:

(14) $$\begin{array}{c} L_{2}=r_{2}-r_{b}=r_{b}\left[{\left(\frac{\mu P_{m}}{\left(1-\mu \right)\left(\sigma_{dt}-\sigma_{\theta \theta geo}\right)}\right)}^{1/\alpha }-1\right]. \end{array}$$

It can be seen from the above points that the loose amount of coal and rock blasting under the action of the blasting wave of the liquid carbon dioxide phase change gas not only affects the liquid in the cracking device, but also is related to the mechanical action and the in-situ stress of the coal body [16].

### 3.2. Numerical Simulation

Stress wave and shock wave propagate in a coal medium with the law of negative exponential attenuation, and the effect of the control hole is different under high stress and in-situ stress [17]. According to the laboratory measurement, when the in-situ stress is 10 MPa, the effective influence radius after single borehole fracturing blasting is 6 m in the direction of air outlet and 4 m in the normal direction. During the numerical simulation, the spacing between CO_2_ crack generators is 10 m and the spacing between the blasting holes is 12 m, and a control hole is set at the midpoint of the two crack holes to increase the free surface [18]. The structural characteristics of FLAC3 porous liquid CO_2_ fracturing blasting are shown in Table 1. The blasting and control holes are set up on time, and the top design method is adopted, and the gravitational pressure of the covering soil of 10 MPa is evenly distributed.

Due to the Hopkinson effect, the shock wave and stress wave are constantly reflected around the control hole, resulting in the superposition of the stress around the borehole. Therefore, a good permeability enhancement and pressure relief effect is formed around the borehole, increasing the area of the fracture area. Therefore, the fragmentation degree of liquid CO_2_ with control holes after blasting is greater than that without control holes. The in-situ stress of 10 MPa is set, the size of the model is 40 × 50 × 5 m^3^, 80000 grids are divided, and there are 89991 nodes in total [19]. Three groups of parameters with different blasting barrel spacing and blasting hole spacing are used for simulation, which are 8 m × 10 m, 6 m × 8 m, and 5 m × 7 m, respectively. The physical and mechanical properties of the model are shown in Table 2.

When the distance between the blasters are 10 m and 12 m, respectively, there is a blank area between the two adjacent blasting holes after blasting, which fails to achieve the antireflection effect. If the distance between the blasters and the distance between the blasting holes is reduced, the blasting areas will be superimposed on each other, the blasting capacity will be significantly weakened, and the blasting cost will be significantly increased. At the same time, the increase of blasting will seriously break the coal body, and the mining of the working face will be affected [20]. When the blasting parameter is 8 m × 10 m (distance between blasters and blasting holes), the blasting effect is not ideal. When the blasting parameter is 6 m × 8 m, the effective radius of blasting increases obviously, but there are still some blank areas that cannot achieve the effect of antireflection. When the blasting parameter is 5 m × 7 m, all areas around the blasting holes are within the CO_2_ effective blasting area, and good blasting effect is achieved [21].

## 4. Results and Analysis

### 4.1. Analysis of Calculation Results

The explosion stress wave is centered on the blast hole and propagates around in the form of concentric circles, and the stress wave energy is gradually attenuated. In order to facilitate comparison, the stress time history curve data of the unit corresponding to the AE of the measuring point are derived in the postprocessing and drawn into Figures 2 and 3. It can be clearly seen that the gas pressure has a significant impact on the coal blasting. Near the blast hole, the gas pressure significantly increases the peak value of the explosion stress wave, as shown in Figure 2. Under the disturbance of blasting dynamic load, the dynamic balance in the coal body is broken. Before the explosion stress wave reaches the measuring point unit, the measuring point unit is subjected to the same pressure as that in the *x*-axis direction, so it shows tensile stress in the *x*-direction stress diagram. After the explosion stress wave reaches the measuring point unit, the gas pressure and explosion stress wave act together to rapidly increase the stress of the measuring point unit and increase the peak stress when there is no gas pressure [22].

The stress time history curve of whether there is gas pressure in the unit at measuring point B far away from the blast hole. As can be seen from Figure 3, due to the high oil content, there is a certain impact on the blasting effect of coal. In the middle and far area of blasting, the peak stress increases in varying degrees and the action time increases slightly. Similarly, due to the blasting action, the dynamic balance of gas pressure is broken, and the unit at measuring point B is affected by the changing force. Therefore, it is shown as a sawtooth curve on the *x*-direction stress curve. The gas pressure is applied in the calculation model, and the blasting stress wave changes in varying degrees. For the blasting effect of coal, the effective energy of explosives can be more fully utilized, and the utilization rate of explosives will increase [23]. The numerical simulation results show that the blasting effect of coal is not only the joint action of the blast stress wave and the blasting gas, but also the gas pressure also participates in the blasting of the coal, and the gas pressure plays an active role in the blasting of the coal, which is beneficial to improve the blasting effect, which is different from rock blasting.

### 4.2. Investigation on Fracture and Permeability Enhancement Effect Caused by Phase Change Gas Explosion in Mining Face

Due to the design experiment to increase the permeability of open-pit mining through phase change gas explosion, two carbon dioxide phase change gas explosion-proof cracks were used in the whole process to try to work. The equipment is mzl300-63/1000, which is independently developed by a research institute, and the explosion relief valve is 200 MPa. The water used for hole sealing is a bag type hole sealing system. According to the measured width of predrainage gas zone in the coal roadway of the experimental working face, the depth of blasting hole sealing is 16 m. After the gas explosion connection is completed, the blasting shall be started from a long distance. No person is allowed to work in the downwind direction of the blasting hole. Surface blasting can be performed 30 minutes after blasting is completed. After the designed borehole completes the liquid carbon dioxide phase change gas cracking and permeation enhancement test, the blasting borehole should be closed and the tracer gas SF6 should be injected immediately after the drilling rig takes out the fracturing device. The extraction borehole (investigation borehole) that has been sealed before blasting shall be connected with the grooved branch pipeline for negative pressure extraction, and then the volume fraction of tracer gas SF6 in the extracted mixed gas shall be monitored in real time in each extraction borehole.

To determine the displacement radius, the tracer fuel method is used. According to the measurement results of this method, it can be seen from Figure 4 that after the coal seam test was blasted and detonated with liquid carbon dioxide phase change oil, the oil tracer was observed at 1.0 m from the stope to increase permeability. Three days after the gas explosion, the wellbore exploded. The measurement results of the gas extraction radius of the original coal show that the tracer gas is monitored for 16 days when it is 1.0 m away from the gas injection borehole, indicating that the phase change gas explosion effectively improves the formation and expansion of fractures within the influence range. From the figure, it can be concluded that the extraction borehole 2 can continuously monitor the tracer gas, while the extraction borehole 3 cannot monitor the tracer gas. Thus, it can be determined that the penetration radius into the radius caused by the carbon dioxide phase transition gas is 2.0 m, which makes it more cost effective for the original gas extraction. The original gas extraction radius of coal seam is effectively increased by 2 times [24]. After the completion of liquid carbon dioxide phase change gas explosion, coal seam drilling is constructed according to the drilling diagram to investigate and test the characteristic coefficient of natural gas emission. The experimental results of coal seam drilling after gas explosion are shown in Figures 5 and 6.

By comparing the carbon emission characteristic curves of coal seam drilling difference , it can be seen that the drilling distance is 1 m and 2 m from the blasting hole, the initial fuel emission of the drilling is 0.6035 m^3^/min-hm and 0.3021 m^3^/min-hm, respectively, and the gas carbon monoxide emission. The attenuation coefficients are 0.023/d and 0.028/d, respectively. Before blasting, the initial gas emission from 100 m drill hole of the original coal body is 0.0746 m^3^/min-hm, and the attenuation coefficient of natural gas emission is 0.031/d. Through the analysis of the above data, it can be concluded that the coalbed methane explosion increases the gas emission of the test borehole 1 m away from the blasting borehole by 8 times, and the attenuation coefficient of gas emission decreases by 0.76 times. The test drilling distance of 2 m from the blasting hole increased the exhaust gas discharged from the borehole by 4 times, and the gas emission attenuation coefficient decreased by 0.93 times, but the gas emission attenuation coefficient did not change. According to the carbon emission characteristic coefficient of coal seam drilling after gas explosion, the optimal gas explosion permeability can be determined as 2 m. The gas flow of the test borehole 3 M away from the blasting borehole increased briefly, but then decreased to the gas emission intensity of the original coal body. It is analyzed that the reason is that the blasting vibration affects the 3 M position, but the crack affected by the vibration closes rapidly under the action of in-situ stress. It can also be seen from the test data that the gas explosion can promote the development of the original fractures of the coal body and form new fractures, connect the fractures, and form a fracture network, so as to improve the gas emission in the borehole. Also, the attenuation coefficient is related to the desorption speed of the coal body itself, which also explains that the gas flow in the borehole increases greatly within the influence range of the gas explosion, but the gas attenuation coefficient decreases slightly.

When selecting an antiseepage device to improve the permeability of deep low-permeability coal seams and high-gas coal seams, the most economical and appropriate antiseepage technology should be adopted in combination with the characteristics of mining connections used in conjunction with the mine's mining connections and the occurrence characteristics of the mine's coal seam. This paper proposes to carry out comparative experimental research on different antireflection technologies in the same mining face, and obtains the antireflection effect and applicability parameters of the corresponding antireflection technologies. During the experiment in the experimental working face, the data analysis results of four aspects of different antireflection technologies are counted: benefit (cost for completing a group of 100 m antireflection measure holes), efficiency (time for completing a group of 100 m antireflection measure holes), effect (antireflection radius), and safety (safety in the process of antireflection). There is the possibility of explosion rejection in deep hole shaped charge blasting, which is easy to cause personal injury in the process of manual recovery or coal mining. At the same time, there is an open fire in the blasting process, which will cause the risk of gas explosion or coal combustion; The explosives and PVC pipes used in deep hole shaped charge blasting are primary consumables and expensive. The preparation time of borehole sealing and related processes of bedding hydraulic fracturing in coal mine is long, the related processes of hydraulic fracturing are complex and the cost of single hole is high. The main consumable of liquid carbon dioxide phase transfer gas is waste carbon dioxide, heating body, and explosion relief valve plate from the chemical plant. The blasting drill is taken out after the use of the cracker and can be used for subsequent blasting drilling. The main cost lies in the cost of purchasing the cracker in the early stage. Since carbon dioxide phase transfer is a safe technique, there will be no safety problem. The high efficiency of this technology is reflected in that after the blasting drilling of this coal seam is completed, the crack generator can be placed into the target drilling hole, and can be taken out after the gas explosion is completed. The whole blasting process can be completed within 8 hours in a small work shift. Based on the above analysis, the optimal antireflection technology can be selected in combination with the actual situation of the mine in the process of engineering practice.

## 5. Conclusion

Based on the finite element dynamic analysis software, the blasting effect of coal is numerically simulated in this paper. The influence of coupled and uncoupled charge structure and gas pressure on coal blasting is analyzed. Through the blasting experiment of coal similar materials, the correctness of the numerical simulation analysis results and the rationality of the modeling are verified. By applying a high oil pressure of 0.7 MPa to the coal body, as a mathematical simulation of the blasting process, it is determined that the coal body has high oil content, which plays a positive role in the development and adjustment of the blasting effect on the coal body. The peak value of the blasting stress wave in the blasting area increases significantly, and the oil pressure strength in the blasting distance is also obvious; in the whole blasting process, the oil pressure increases the peak rate of the wave stress and delays. The rapid decay of the stress wave prolongs the duration of the stress wave. It shows that the blasting effect of coal is not only the combined effect of explosion stress wave and gas explosion, but also the result of the combined effect of explosion stress, high wave, explosion, and gas. The comparative experimental results of three groups of different antireflection technologies in mining show that the influence range of antireflection measures on coal body is: hydraulic fracturing > deep hole shaped charge blasting > liquid carbon dioxide phase change gas explosion. The maximum oil volume fraction of the extractor is: liquid carbon dioxide phase change oil explosion > deep blasting rate > hydraulic fracturing; the oil attenuation coefficient in the well is: liquid carbon dioxide phase change oil explosion < hydraulic fracturing≤ deep blasting equivalent. At the same time, the comparative experiment also quantifies the benefit, efficiency, effect, and safety indexes of different antireflection technologies in the field implementation process. The mechanism of coal blasting and the dynamic response of surrounding coal is a very complex research topic. Under the condition that the current theoretical research is not very sufficient, it is an effective method to use the powerful numerical calculation software to calculate and analyze the coal blasting process, which is conducive to promote the research of the theory of coal blasting.

## Figures and Tables

**Figure 1:** Air source protection system.

**Figure 2:** Stress time history curve in the *X* direction at measuring point A.

**Figure 3:** Stress time history curve in the *X* direction at measuring point B.

**Figure 4:** Variation curve of tracer gas volume fraction in experimental pumping boreholes with gas burst antireflection radius.

**Figure 5:** Attenuation curve of gas emission from the test borehole (1 m from the blasting hole).

**Figure 6:** Attenuation curve of gas emission from the test borehole (2 m from the blasting hole).

**Table 1:** Basic parameters of coal seam.

Parameter	Calculation area/m^3^	Crack hole diameter/m	Number of grids/piece	Number of nodes/piece	Applied overburden self-weight stress/MPa
Numerical value	52 × 60 × 5	0.1	124500	136824	10

**Table 2:** Mechanical parameters of the model.

Bulk density/kg∙m^−3^	Bulk modulus/GPa	Shear modulus/GPa	Internal friction angle/°	Cohesion/MPa	Uniaxial tension/MPa
1350	1.51	0.57	39	1.4	0.58

## Data Availability

The data used to support the findings of this study are available from the author upon request.
